This article has been retracted.

# Establishment of Difficult Caudal Epidural Blockade Prediction Model

**DOI:** 10.1155/2022/2037904

**Published:** 2022-11-04

**Authors:** Guohao Xie, Jialian Zhao, Lihua Chu, Shengwen Song, Ya Wang, Dengming Lai, Baoli Cheng, Xiangming Fang

**Affiliations:** ^1^Departments of Anesthesiology, The First Affiliated Hospital, School of Medicine, Zhejiang University, Hangzhou, Zhejiang, China; ^2^Departments of Anesthesiology, The Children's Hospital, School of Medicine, Zhejiang University, Hangzhou, Zhejiang, China; ^3^Departments of Neonatal Surgery, The Children's Hospital, School of Medicine, Zhejiang University, Hangzhou, Zhejiang, China

## Abstract

**Background:**

We aimed to develop a predictive difficult caudal epidural blockade (pDCEB) model when ultrasound was not available and verified the role of ultrasound in difficult caudal epidural blockade (CEB).

**Methods:**

From October 2018 to March 2019, this study consisted of three phases. First, we prospectively enrolled 202 patients scheduled to undergo caudal epidural anesthesia and assessed risk factors by binary logistic regression to develop the predictive scoring system. Second, we enrolled 87 patients to validate it. The receiver operating characteristic (ROC) curve was used to evaluate the performance of the prediction model. Youden-index was used to determine the cut-off value. Third, we enrolled 68 patients with a high risk of difficult CEB (pDCEB score ≥3) and randomized them into ultrasound and landmark groups to verify the role of ultrasound.

**Result:**

The rate of difficult CEB was 14.98% overall 289 patients. We found a correlation between unclear palpation of the sacral hiatus (OR 9.688) and cornua (OR 4.725), the number of the sacral hiatus by palpation ≥1 (OR 4.451), and history of difficult CEB (OR 39.282) with a higher possibility of difficult CEB. The area under the receiver operating characteristic curve of the pDCEB model involving the aforementioned factors was 0.889 (95% CI, 0.827–0.952) in the development cohort and 0.862 (95% CI, 0.747–0.977) in the validation cohort. For patients with a pDCEB score ≥3, a preprocedure ultrasound scan could reduce the incidence of difficult CEB (55.56% in the Landmark group vs. 9.38% in the ultrasound group, *p* < 0.001).

**Conclusion:**

This novel pDCEB score, which takes into account palpation of the sacral hiatus/cornua, number of the sacral hiatus by palpation ≥1, and history of difficult CEB, showed a good predictive ability of difficult CEB. The findings suggested that performing an ultrasound scan is essential for patients with a pDCEB score ≥3. Trial registration: No: ChiCTR1800018871, Site URL: https://www.chictr.org.cn/edit.aspx?pid=31875&htm=4; Principal investigator: Jialian Zhao, Date of registration: 2018.10.14.

## 1. Introduction

Caudal epidural blockade (CEB) is one of the most common techniques performed on pediatric patients [1, 2]. Moreover, it is used in several adult surgical techniques, such as prostate biopsy [3], anorectal surgery [4], and treatment of lumbar spinal disorders or chronic back pain [5]. Compared with other neuraxial techniques, such as spinal or epidural blocks, caudal blocks are rarely associated with hypotension and bradycardia, given their lower sympathetic blockade [1]. This indicates that CEB may have advantages in patients with advanced cardiac disease or other diseases [6, 7]. Performing a CEB is simple and easy to learn; however, a rate as high as 25% of incorrect needle placements, even with experienced anesthesiologists, has been reported in several patients [8]. Like other neuraxial blockades, CEB difficulties are mainly associated with the quality of palpable surface landmarks [9–11]. Successfully performing a CEB mainly depends on the accurate identification of the sacral hiatus, which is usually easily palpable but with considerable anatomical variations. Up to now, there is still no predictive assessment protocol for difficult CEB in adult patients.

The ultrasound technique has been applied to improve peripheral nerve blockade and central neuraxial interventions [12–14]. It can be used to provide sonographic images that show anatomical variations of the sacral hiatus, which is currently regarded as a gold standard for correct needle placement in the CEB technique [15, 16]. However, ultrasound-guided CEB may not be available in resource-limited regions/hospitals and needs much more experience and ultrasound technique of anesthetists. In many hospitals in developing countries or regions, there was only one or even no ultrasound device in the department of anesthesiology. It is only recommended in cases where anatomical detection of the sacral hiatus is difficult, especially via palpations [17–19]. Therefore, it is necessary to develop a scoring model for difficult CEB using surface anatomical landmarks and clarify the role of ultrasound to the clinical anesthetists in cases of a difficult caudal epidural block (DCEB).

We took advantage of new statistical methodologies that incorporated machine and deep learning into prediction models to develop an objective risk scoring model, which is widely used in predicting the evolution of the disease in patients or the risk of mortality in patients [20, 21]. We hypothesized that palpation and other objective factors can predict difficult CEB well. Thus, we aimed to assess the risk factors for DCEB and develop a predictive difficult caudal epidural block (pDCEB) scoring system based on the surface anatomical landmarks and other factors. In addition, we aimed to determine whether a pre-procedure ultrasound scan can facilitate the CEB procedure in these patients.

## 2. Methods

### 2.1. Study Design and Participants

This prospective study was carried out at the First Affiliated Hospital of Zhejiang University (Hangzhou, China) after being approved by the local Ethics Committee and registered in the Chinese Clinical Trial Registry (ChiCTR1800018871, site URL: https://www.chictr.org.cn/edit.aspx?pid=31875&htm=4). Written informed consents were obtained from the patients or their authorized legal representatives. We enrolled patients undergoing anorectal surgery and scheduled to undergo caudal epidural anesthesia with an American Society of Anesthesiologists (ASA) physical status of I–II. We excluded patients with sacrococcygeal diseases such as spinal meningocele, teratoma, and infection, with coagulation defects, or refusing caudal epidural anesthesia.

From October 31^st^, 2018, to March 31^st^, 2019, we enrolled a total of 375 patients scheduled for anorectal surgery in three phases. In the development cohort (phase one), we included 215 patients, among whom we excluded 13 patients with teratoma (*n* = 1), coagulation defects (*n* = 6), infection at the puncture site (*n* = 2), and those who refused CEB (*n* = 4). In the validation cohort (phase two), we included 90 patients, among whom we excluded 3 patients according to the exclusion criteria (2 for coagulation defects and one for refusing CEB). We finally included 202 and 87 patients in the development and validation cohort, respectively. In the third phase, we included 70 patients with a pDCEB score ≥3 and included 32 patients in the Ultrasound (Us) group and 36 in the Landmark (Lm) group (Figure 1).

Five senior anesthesiologists with more than five years of CEB experience were arranged to perform the palpation and CEB in the development cohort and three others in the validation cohort. These eight senior anesthesiologists also conduct the third step. An assistant recorded the patients' information, palpation, and the CEB inducer and also assisted the anesthesiologist in performing the ultrasound.

### 2.2. Development of pDCEB

#### 2.2.1. Preparation and Monitoring

Patients were placed in a prone position with the pelvis supported by a pillow and standard monitoring equipment (three-lead electrocardiogram, noninvasive blood pressure, respiratory rate, pulse rate, and pulse oximetry) was implemented. They were administered with 1-2 mg intravenous midazolam for anxiety.

#### 2.2.2. Assessment and Palpation

Before the CEB procedure, the anesthetists palpated the surface landmarks (sacral hiatus and sacral cornua) and recorded the corresponding assessments of the sacral hiatus and cornua. Palpation of the sacral hiatus was classified as either clear/easy to palpate or unclear/difficult to palpate, while the assessment of the sacral cornua was classified as either clear or unclear. Sometimes more than one pit may be palpated in the sacral caudal area. If the number of the “sacral hiatus” by palpation was >1 (more than one pit was palpated in the sacral area), the number was recorded and the anesthetist, based on their experience, would determine an optimal puncture site. Since the palpation and assessment were purely subjective, senior clinical anesthetists experienced at CEB were included to perform in this study to minimize bias.

#### 2.2.3. CEB Procedure

After being sterilized and draped, a 22 G-needle was inserted into the predetermined puncture site. Once there was a loss of resistance and no blood or fluid was aspirated, we placed the sterile ultrasound probe of 13-6 MHz linear array (Sonosite Inc., Bothell, WA, USA or Mindray Inc., Shenzhen, China) transversely to the caudal canal a few centimeters above the needle insertion point. Color flow Doppler imaging was utilized during the actual injection into the caudal epidural space. If the presence of real-time turbulence or color flow within the caudal space during the injection was accompanied by the dilation of the caudal canal (Figure 2(a)), we considered the puncture successful [2, 16, 22] and administered local anesthetics. If the ultrasound indicated the puncture was not successful, the anesthesiologist attempted another puncture until it met the criteria to be successful or failed. After administering a test dose, 10 mg lidocaine (1%) and 7.5 mg ropivacaine (0.375%) were injected into the caudal space. All the palpation, the assessment, and the procedure of CEB were performed by the same anesthetists with more than five years of experience in the caudal epidural blockade.

#### 2.2.4. Data Collection

The duration of the puncture (from the first needle insertion into the skin to the ultrasound confirming the puncture as successful), the number of needle passes (once the needle moves, there was one count of needle passes), the number of attempts (once the needle was withdrawn and new palpation was conducted, there was one count of attempts) during the whole procedure were recorded. DCEB was defined as one where the duration of the puncture was longer than 5 minutes or with more than 10 needle passes or more than 3 attempts, according to the clinical experience and reference [23, 24]. We recorded other objective variables, such as age, Body Mass Index (BMI), a history of DCEB, and a history of sacrococcygeal diseases (fracture, Ankylosing spondylitis, etc.) before the CEB procedure.

### 2.3. Validation of pDCEB

For the validation cohort, all the assessments of the surface landmarks and the CEB procedure were similar to those of the development cohort, except for the fact three other senior anesthetists were arranged to perform the palpation and CEB.

### 2.4. Ultrasound for Predicting Patients at Risk of DCEB

We selected a predictive difficult caudal epidural block (pDCEB) score of 3 with the largest Youden-index as the cut-off value, with a score above this being predictive of DCEB. In the Us group (*n* = 32), the patients underwent a preprocedure ultrasound scan to assess the anatomy of the sacral hiatus, sacral cornua, and caudal space, which, together with palpation, was used by the anesthesiologist to determine the puncture site (Figures 2(b) and 2(c)). In the Lm group (*n* = 36), the anesthesiologist palpated the surface landmarks of the sacral hiatus and sacral cornua to determine the puncture site. The rest of the puncture procedure was the same as the above mentioned. The time taken to establish the puncture site (from the start of the preprocedure ultrasound scan/palpation to the start of needle insertion, including sterilizing and draping), duration of the puncture, the total number of needle passes/attempts, the rate of success on the first needle pass, the rate of DCEB, and the patients' satisfaction were recorded.

### 2.5. Statistical Analysis

Quantitative variables were presented as mean ± SD or median (interquartile range, IQR) and analyzed using Student's *t*-test or Mann–Whitney test while categorical variables were presented as *n* (%) and analysed using chi-square test. After above-mentioned univariate analysis, significant variables (*p* value < 0.05) were subjected to binary logistic regression (Forward, LR) to fit the predictive model with an entry level of 0.05 and an exclusion level of 0.10. The goodness of fit of a model was judged using the Hosmer-Lemeshow test and receiver operating characteristic (ROC) curve. An area under the ROC curve (AUROC) > 0.75 was considered to have good predictive ability. Youden-index was used to determine the cut-off value. Patients with a pDCEB score equal or more than 3 were predicted to be at risk of DCEB. All the statistical tests were two sided and performed by SPSS 20.0 software. Nomogram was performed by the software of RStudio (4.1.2). Differences with a *p* value < 0.05 were considered significant.

## 3. Results

### 3.1. Development of the pDCEB

#### 3.1.1. Basic Characteristics and Risk Factors

In the development cohort, the rate of DCEB was 14.85%. There were no significant differences in the patients' basic characteristics regarding gender, age, and BMI. Unclear palpation was much more common in the DCEB cases, including unclear palpation of the sacral hiatus (66.67% vs. 11.63% in the controls, *p* < 0.001) and cornua (73.33% vs. 23.84% in the controls, *p* < 0.001). Patients with DCEB were less satisfied with the procedure. Detailed information is listed in Table 1.

#### 3.1.2. Establishment of the pDCEB Model

Findings of multivariate logistic regression analysis of the predictors of DCEB are listed in Table 2. Unclear palpation of the sacral hiatus (OR, 9.688; 95% CI, 3.323–28.201) and sacral cornua (OR, 4.725; 95% CI, 1.577–14.151), number of the “sacral hiatus” by palpation ≥1 (OR, 4.451; 95% CI, 1.520–13.031), and history of DCEB (OR, 39.282; 95% CI, 2.751–560.827) were correlated with a higher possibility of DCEB. The nomogram of pDCEB is shown in Figure 3.

To meet the objective of developing a simplified model that could calculate the risk of DCEB by simply counting the number of risk factors, we finally rounded off the coefficients. Therefore, we developed the pDCEB and obtained the final score as the summation of the difficulty predictors of each patient (Table 2). The simplified DCEB score is as follows:

The simplified DCEB score = 1.5*∗*More than one “sacral hiatus” by palpation + 4*∗*A history of difficult CEB + 2*∗*Inability or uncertainty to palpate sacral hiatus + 1.5*∗*Inability or uncertainty to palpate the sacral cornua.

ROC was used to evaluate the predictive efficiency of the difficulty score (Figure 4). The AUROC in the development cohort was 0.889 (95% CI, 0.827–0.952; *p* < 0.001). Based on the sensitivity and specificity of the simplified pDCEB score, the cut-off value was 2.5, with the largest Youden-index of 0.628 (sensitivity = 0.733 and specificity = 0.895). Therefore, we selected a score of 3 as the cut-off value, with a score of this and above being indicative of a risk of DCEB.

### 3.2. Validation of the pDCEB

In the validation cohort, the rate of DCEB was 14.94%. There were no significant differences in the patients' basic characteristics, while unclear palpation of the sacral hiatus and cornua, number of the “sacral hiatus” by palpation >1, and history of DCEB were associated with DCEB (Table 1). The AUROC was 0.862 in the validation cohort (95% CI, 0.747–0.977; *p* < 0.001) and showed a good predictive ability (Figure 4).

### 3.3. Ultrasound for Predictive DCEB Patients

In the final phase, we enrolled 68 patients with a pDCEB score ≥3 with no significant difference in the DCEB score among them (Us 3.5 (3.5–5.0) vs. Lm 3.5 (3.5–5.0), *p*=0.736). The DCEB incidence in the Us group was 9.38%, which was significantly reduced compared with the Lm group (55.56%, *p* < 0.001). In the Us group, the number of needle passes and attempts was significantly reduced (2 (1–4) vs. 9 (3–15), *p* < 0.001; 1 (1-2) vs. 3 (1.25–5), *p* < 0.001), and the success rate on first needle pass was significantly increased (46.88% vs. 8.33%, *p* < 0.001), and the time to perform CEB was significantly reduced (1 (1–2.75) vs. 6 (2–7.75), *p* < 0.001). Moreover, the Us group needed more time to establish the puncture site, but there was a significant between-group difference in the total procedure (both *p* < 0.001). Patients in the Us group were more satisfied with the anesthesia. There was no significant between-group difference in the use of a rescue analgesia drug (Table 3).

## 4. Discussion

This prospective study demonstrated that unclear palpation of the sacral hiatus and sacral cornua, number of the “sacral hiatus” by palpation ≥1, and history of DCEB were the four predictors of DCEB. We developed the pDCEB score and found that the ROC in the two cohorts both showed good predictive ability. All the patients were stratified into a score range of 0–9, with a score of 3 as the cut-off value. For patients with a pDCEB score ≥3, ultrasound-assisted CEB reduced the number of needle passes and the duration of the puncture duration and improved the rate of successful punctures on the first needle pass and the patients' satisfaction.

Palpation of the sacral hiatus was the main factor in determining the difficulty during the caudal epidural injection. Unlike other neuraxial techniques, such as spinal and epidural anesthesia, age and obesity were not correlated with DCEB, which may be due to the superficial anatomical structure of sacral hiatus and the operation of this procedure [4, 25]. Studies have shown that the distance between the skin and the posterior sacral bony surface is 17.5 ± 4.7 mm and that the distance between the bilateral cornua was 18.1 ± 3.2 mm with ultrasonographic evaluation [26]. There can be considerable variations in the heights and shapes of the sacral hiatus depending on the developmental fusion processes of the sacral vertebrae and ligaments during childhood [2, 22, 27]. In most people, the sacral hiatus is formed by incomplete fusion of the S5 vertebrae in the posterior mid-line. However, some patients also show an incomplete fusion of the lower portion of the S4, S3, or S2 posterior mid-line [2]. In a few cases, the hiatus has been reported to be absent in the fusion processes or the sacrococcygeal membrane and cannot be penetrated because of advanced ossification, which has resulted in the failure of CEB [28]. We also found that the sacral cornua, formed by the remnants of the S5 inferior articular processes, are significantly associated with caudal epidural anesthesia in this study. However, there have been reports of the sacral cornua being impalpable or unilateral in up to 46% to 79% of cases [8, 25], thus causing the clinical anesthesiologist difficulty. We found that more than one “sacral hiatus” by palpation was a predictor of DCEB, which might be due to the fake hiatus between the median sacral crest or irregular variations.

A successful CEB depends on the accurate placement of the needle into the caudal epidural space; however, there was a certain incorrect needle placement rate even with experienced anesthesiologists [2, 27]. With advances in medical imaging, fluoroscopy, computed tomography (CT), magnetic resonance imaging (MRI), and ultrasound can all be used to reveal the anatomy of the sacral hiatus and assist the anesthesiologist while performing the CEB [29–31]. Preprocedural ultrasound scanning was reported to facilitate spinal anesthesia by allowing appropriate selection of the intervertebral space, needle alignment, measuring the depth from the skin to dura, reducing the number of attempts, and decreasing the number of bony contacts and associated complications in adult patients with difficult surface anatomic landmarks [23, 32]. Compared with the conventional blind method, ultrasonography can allow one to visualize the anatomic structure of the sacral hiatus and the spread of the local anesthetics [2, 15, 16, 33]. Ultrasonography has been reported to be superior to the “swoosh” test as an objective confirmatory technique during caudal block placement and allows 100% accuracy in correct needle placement [15, 34, 35]. Based on this, we chose ultrasound to allow and determine successful punctures. To avoid the influencing factor of the practicing anesthesiologist, we placed the ultrasound probe a few centimeters cephalad to the point of needle insertion and checked for whether there was accompanying real-time turbulence or color flow within the caudal space during injection with dilation of the caudal canal.

Ultrasound is a valuable tool for identifying anatomical landmarks of the sacral hiatus in CEB [26, 36, 37]. Compared with the conventional landmark technique, preprocedural ultrasound or ultrasound-guided CEB conferred superior advantages since it allows real-time visualization of the anatomical structures and spread of the local anesthetic [16, 19, 34]. We found that ultrasound reduced the DCEB rate and the total number of needle passes/attempts and increased the success rate on the first needle pass. This might indicate that the traditional landmark-based method should be abandoned. But in resource-limited regions/hospitals, an ultrasound may not be available for every anesthetist and it also asks for much more experience and ultrasound technique. In many hospitals in developing countries/regions, there is only one or even no ultrasound in the anesthesiology department. Also, ultrasound was not suggested for every patient since its high success rate. In pediatric patients, studies have suggested that ultrasound is only essential if the sacral cornua and sacral hiatus are clinically identifiable [19, 38]. In our study, the DCEB rate in the 287 patients was 14.88%, while those with a low DCEB score (DCEB score <3) had a DCEB rate as low as 5.19%. This indicates that ultrasound assistance is not needed for patients with low DCEB scores (DCEB score <3). Moreover, given the superficial anatomical structure of the sacral hiatus, there was no significant difference between preprocedure ultrasound and ultrasound-guided CEB.

There are several limitations to this study. One is that the development and validation of this predictive scoring system were both conducted in a single center. Thus, multicentre studies should be conducted to improve and validate this predictive scoring system for DCEB. The other is that all palpation and assessments of the sacral hiatus area were purely subjective. Even though experienced senior clinical anesthetists performed the CEB procedure, this could still have resulted in bias.

## 5. Conclusions

Palpation of the sacral hiatus structures, including the sacral hiatus and sacral cornua, number of the “sacral hiatus” by palpation ≥1, and history of DCEB, were risk factors associated with DCEB in adult patients. The preoperative score consisting of these four factors showed good predictive ability. Our findings indicated that ultrasound is suggested only in a higher risk of DCEB (pDCEB score ≥3) cases in order to save resources and cost, especially in resource-limited regions/hospitals.

## Figures and Tables

**Figure 1:** From October 31^st^, 2018, to March 31^st^, 2019, we enrolled a total of 377 patients scheduled for anorectal surgery in three phases. In the development cohort (phase one), we included 215 patients were included, among whom we excluded 13 patients with teratoma (*n* = 1), coagulation defects (*n* = 6), infection at the puncture site (*n* = 2), and those who refused CEB (*n* = 4). In the validation cohort (phase two), we included 90 patients, among whom we excluded 3 patients were excluded according to the exclusion criteria (2 for coagulation defects and one for refusing CEB). We finally included 202 and 87 patients in the development and validation cohort, respectively. In the third phase, we included 72 patients with a pDCEB score ≥3 and finally included 32 patients in the Ultrasound (Us) group and 36 in the Landmark (Lm) group after exclusion.

**Figure 2:** Colour flow Doppler imaging of a “successful puncture” (a). Ultrasound images of the transverse (b) and longitudinal (c) plane of the sacral hiatus. Real-time turbulence or color flow and expansion of the caudal space during an injection can be seen. The area of turbulence or color flow is the caudal space. The “white triangle” represents the sacral cornua, the “downward arrow” represents the sacrococcygeal ligament, the “leftward arrow” represents the base of the sacrum posterior surface, and the “double-ended arrow” represents the caudal space.

**Figure 3:** Nomogram of the pDCEB. The “Points” represents the single item score corresponding to each variable, while the “Total points” represents the sum of the individual scores corresponding to the values of all variables. The “prob of DCEB” is the risk of difficult caudal epidural blockade.

**Figure 4:** ROC curves based on the DCEB scoring model and its respective AUROC (95% CIs). The blue solid curve is the ROC curve from the development cohort (*n* = 202), while the dotted curve represents the validation cohort (*n* = 87). The ROC curve was used to evaluate the efficiency of prediction and an area under the ROC curve (AUROC) > 0.75 is considered to indicate a good predictive ability.

**Table 1:** Basic characteristics of the development and validation cohort.

Characteristics	Development cohort *N* = 202			Validation cohort *N* = 87		
*N* = 289	DCEB (*N* = 30)	No DCEB (*N* = 172)	*p* Value	DCEB (*N* = 13)	No DCEB (*N* = 7)	*p* Value
Male	22 (73.33%)	127 (73.84%)	0.954	11 (84.62%)	49 (66.22%)	0.186
Age	45.10 ± 14.08	41.82 ± 14.73	0.249	41.69 ± 11.93	4.22 ± 13.85	0.898
BMI	23.67 ± 3.72	23.43 ± 3.41	0.747	24.85 ± 3.76	22.43 ± 3.15	0.045^*∗*^
A history of difficult CEB	3 (10.00%)	1 (0.58%)	0.011	2 (15.38%)	0 (0.00%)	0.001^*∗*^
Distance between puncture site and coccygeal apex (cm)	6.5 (6.0–7.125)	6.5 (6.0–7.0)	0.855	7.5 (7–8)	7 (6.875–7.5)	0.253
Number of “sacral hiatus” by palpation			0.006			0.001^*∗*^
1	17 (56.67%)	141 (81.98%)		6 (46.15%)	57 (77.03%)	
2	10 (33.33%)	26 (15.12%)		3 (23.08%)	15 (20.27%)	
≥3	3 (10.00%)	5 (2.90%)		4 (30.77%)	2 (2.70%)	
Unclear palpation of sacral hiatus	20 (66.67%)	20 (11.63%)	<0.001^*∗*^	6 (46.12%)	5 (6.76%)	<0.001^*∗*^
Unclear palpation of sacral cornua	22 (73.33%)	41 (23.84%)	<0.001^*∗*^	9 (69.23%)	16 (21.62%)	<0.001^*∗*^
Patient and surgeon satisfaction			<0.001^*∗*^			<0.001^*∗*^
Very satisfied	15 (50.00%)	153 (88.95%)		5 (38.46%)	71 (95.95%)	
Satisfied	6 (20.00%)	17 (9.88%)		5 (38.46%)	2 (2.70%)	
Dissatisfied	9 (30.00%)	2 (1.16%)		3 (23.08%)	1 (1.35%)	
Success on 1st needle pass	0 (0.00%)	91 (45.05%)		0 (0.00%)	40 (47.06%)	—

BMI: Body Mass Index; CEB: Caudal Epidural Blockade/Block. The values are presented as mean ± standard deviation (SD), median (interquartile range, IQR), or *n* (%). Normally distributed continuous variables are presented as “Mean ± SD” while abnormally distributed ones are presented as “Median, IQR”. Categorical variables are presented as “*n* (%),” Each ^*∗*^*p* value < 0.05 was considered to be significant. The *p* value was obtained by Student's *t*-test or Mann-Whitney test for continuous variables and chi-square test for categorical variables.

**Table 2:** Risk factors associated with difficult caudal epidural block and the simplified model of pDCEB score.

Covariants	*β* coefficient	OR	Or 95% CI	*p* Value	Point
Unclear palpation of sacral hiatus	2.271	9.688	3.323–28.201	<0.001	2
A history of difficult CEB	3.671	39.282	2.751–560.827	0.007	4
Unclear palpation of sacral cornua	1.553	4.725	1.577–14.151	0.006	1.5
More than one sacral hiatus	1.493	4.451	1.520–13.031	0.006	1.5
Constant	−3.911	0.02	—	<0.001	—

Hosmer–Lemeshow test *p*=0.732. The risk was calculated using odds ratio [OR] (confidence interval [CI]). Each *p* value < 0.05 was considered significant. All the variants entered into the regression analysis were categorical: more than one sacral hiatus by palpation indicated 1 while only one sacral hiatus by palpation indicated 0; a history of difficult CEB indicated 1; inability to palpate or uncertain feeling of the sacral hiatus indicated 1 while clear palpation of the sacral hiatus indicated 0; inability to palpate or uncertain feeling of the sacral cornua indicated 1 while clear palpation of the sacral cornua indicated 0. We used binary logistics regression (Forward, LR) to fit the model with an entry level of 0.05 and an exclusion level of 0.10. The simplified DCEB score = 1.5^*∗*^. More than one “sacral hiatus” by palpation +4^*∗*^. A history of difficult CEB +2^*∗*^. Inability or uncertainty to palpate sacral hiatus +1.5^*∗*^. Inability or uncertainty to palpate the sacral cornua.

**Table 3:** Performance of CEB between the ultrasound and landmark group in predictive DCEB patients (DCEB score ≥3).

	Ultrasound group (*N* = 32)	Landmark group (*N* = 36)	*p* Value
DCEB score	3.5 (3.5–5.0)	3.5 (3.5–5.0)	0.736
Difficult CEB	3 (9.38%)	20 (55.56%)	<0.001^*∗*^
Success on 1st needle pass	15 (46.88%)	3 (8.33%)	<0.001^*∗*^
Time take to establish puncture site	7 (6–8)	3 (2.25–4.0)	<0.001^*∗*^
Time take to perform CEB	1 (1–2.75)	6 (2–7.75)	<0.001^*∗*^
Total procedure time	9 (7–10.75)	9 (5–11)	0.308
Total number of needle passes	2 (1–4)	9 (3–15)	<0.001^*∗*^
Total number of attempts	1 (1–2)	3 (1.25–5.0)	<0.001^*∗*^
Rescue analgesia drug	5 (15.63%)	10 (27.78%)	0.228
Patient's satisfaction			<0.001^*∗*^
Satisfied	28 (87.5%)	17 (47.22%)	
Qualified	2 (6.25%)	15 (41.67%)	
Dissatisfied	2 (6.25%)	4 (11.11%)	

The values are presented as mean ± standard deviation (SD), median (interquartile range, IQR), or *n* (%). Normally distributed continuous variables are presented as “Mean ± SD” while abnormal distributed ones are presented as “Median, IQR.” Categorical variables are presented as “*n* (%).” Each ^*∗*^*p* value < 0.05 was considered significant. The *p* value was obtained by Student's *t*-test or Mann-Whitney test for continuous variables and chi-square test for categorical variables.

## Data Availability

Data from the reported cases will be made available on reasonable request from the corresponding author.
